RETRACTED

# Genome-wide investigation and functional analysis of RNA editing sites in wheat

**DOI:** 10.1371/journal.pone.0265270

**Published:** 2022-03-11

**Authors:** Fatima Rasool, Iqra Ishtiaq, Muhammad Uzair, Ali Ahmed Naz, Jens Léon, Muhammad Ramzan Khan

**Affiliations:** 1 Genome Editing & Sequencing Lab, National Centre for Bioinformatics, Quaid-i-Azam University, Islamabad, Pakistan; 2 National Institute for Genomics and Advanced Biotechnology, National Agriculture Research Centre, Park Road, Islamabad, Pakistan; 3 Institute of Crop Science and Resource Conservation (INRES), Department of Crop Genetics and Biotechnology, Rheinische Friedrich-Wilhelms University of Bonn, Bonn, Germany; The University of Haripur, PAKISTAN

## Abstract

Wheat is an important cereal and half of the world population consumed it. Wheat faces environmental stresses and different techniques (CRISPR, gene silencing, GWAS, etc.) were used to enhance its production but RNA editing (RESs) is not fully explored in wheat. RNA editing has a special role in controlling environmental stresses. The genome-wide identification and functional characterization of RESs in different types of wheat genotypes was done. We employed six wheat genotypes by RNA-seq analyses to achieve RESs. The findings revealed that RNA editing events occurred on all chromosomes equally. RNA editing sites were distributed randomly and 10–12 types of RESs were detected in wheat genotypes. Higher number of RESs were detected in drought-tolerant genotypes. A-to-I RNA editing (2952, 2977, 1916, 2576, 3422, and 3459) sites were also identified in six wheat genotypes. Most of the genes were found to be engaged in molecular processes after a Gene Ontology analysis. *PPR* (*pentatricopeptide repeat*), *OZ1* (*organelle zinc-finger*), and *MORF/RIP* gene expression levels in wheat were also examined. Normal growth conditions diverge gene expression of these three different gene families, implying that normal growth conditions for various genotypes can modify RNA editing events and have an impact on gene expression levels. While the expression of *PPR* genes was not change. We used Variant Effect Predictor (VEP) to annotate RNA editing sites, and Local White had the highest RESs in the CDS region of the protein. These findings will be useful for prediction of RESs in other crops and will be helpful in drought tolerance development in wheat.

## Introduction

RNA editing was discovered 30 years ago. RNA editing is a post-transcriptional variation of transcripts encoded by the chloroplast, nucleus, or mitochondrial genome of animals and plants, and it was first reported in protozoan mitochondria and then in plant [1–4]. RNA molecules are covalently modified by RNA editing process in eukaryotes, resulting in substitutions, deletions of amino acids and variations in expression levels of genes, including changes in protein diversity [5–9]. In plant organellar transcripts, it was previously thought to be an error-correcting process. On the other hand, the current sequence resources of genomes and transcriptome enabled researchers to better comprehend its importance in plants developments under the abiotic stress conditions [10]. The most common editing types in non-flowering land plants are adenosine (A) to inosine (I) in tRNA, cytidine (C) to uridine (U) in messenger tRNA and RNA, and urea to cytidine (C) in mRNA [11]. The RNA editing in plants is important because as certain mutants with poor editing died at early stage of development [11]. Protein function at the RNA level is maintain by RNA editing events, e.g., failure of editing of the plastid ATPase alpha-subunit mRNA causes the pigment deficiency in tobacco cybrids [12]. In plants, the *pentatricopeptide repeat* (*PPR*) family is responsible for cytidine (C)-to-uridine (U) editing, whereas in mammals, adenosine deaminase is responsible for adenosine (A) to inosine (I) editing (ADAR). RNA editing is a fundamental factor in primate evolution, and it plays a crucial function in regulating environmental stress. Previous study has revealed the wide range of adenosine (A) to inosine (I) editing in mammalian transcriptomes that are involved in biological processes such as nervous system development [13, 14].

RETRACTED

The identification of RNA editing targets is an important first step in gaining a deeper understanding of this post-transcriptional modification and entire genome and transcriptome sequence of the same individual to exclude polymorphisms and mutations between populations, including experimental methods with the necessary high-throughput sequencing and background resolution are required [15, 16]. Deep transcriptome sequencing such as RNA-Seq can examine the entire transcriptome at once, making it a valuable tool in this field [17–19]. It has been reported that RNA-Seq was used to find wheat RNA editing sites in recent publications, demonstrating that this technique offers advantages in solving many unsolved problems of editing phenomena, including its impact on the transcriptome.

Wheat (*Triticum aestivum* L.) is a major staple food crop grown in both irrigated and rainfed locations around the world, accounting for 17 percent of arable land and provides important food calories, especially to the 4.5 billion people who live in poor countries [20–22]. Wheat yield is predicted to be reduced by 6.0 percent for every °C rise in global temperature, because of climate variation, as well as more frequent exposure to extended drought periods [22–26]. The scope and consequences of RNA processing by RESs in finding the difference between drought-tolerant and drought-sensitive genotypes remain unanswered until now. Although there are many different types of RESs in the nuclear transcriptome, their impact on drought-sensitive and drought-tolerant wheat genotypes remains unknown. Using entire mRNA deep-sequencing data, we investigated the impact of environmental factors such as drought on RNA processing. More RNA editing events were found in drought-tolerant genotypes, which could be due to high expression of genes in *OZ1* and *MORF/RIP* or RNA editing factor stability. Drought promotes fast RNA editing of the wheat transcriptome, resulting in a shift in the ratio of edited to unedited proteins in the proteome. According to our findings, amino acid alterations in these genes may also play a role in wheat stress adaptation. These key findings tell the story that genetic variation is common, highlighting the significance of a thorough description of these polymorphisms for better understanding wheat growth under normal conditions.

RETRACTED

## Materials and methods

### Plant material and growth conditions

The seeds of drought-sensitive wheat (Batis and Blue Silver) and drought-tolerant wheat (Local White; a land race from dry areas of Pakistan, Chakwal 50, UZ-11-CWA-8, and Syn-22, which is synthetic wheat), were germinated on moist germination paper. After 72 h of germination, four germinated seeds of each genotype were shifted in soiled filled pots consisting of PVC pipes (4.5 cm diameter × 45 cm depth). Each genotype was repeated thrice. Pots were kept at 24/12 ± 2°C Day/night temperature with 10 hours photoperiod in the field. The seedlings were grown under well-watered condition for 35 days. The whole experiment was conducted during wheat growing season in natural conditions. At 35-days-old-seedling stage of wheat, roots samples (each data point pooled from eight plants) were taken as previously described [27, 28] for RNA extraction and sequencing. In details roots of eight plants (35-days-old-seedlings) were pooled and stored immediately in -80°C. This was done to minimize the variation across the samples. Local White, Chakwal 50, and Blue Silver seeds were donated by the Bio-Resource Conservation Institute of the National Agricultural Research Centre in Islamabad. Seeds of Batis, UZ-11-CWA-8, and Syn22 were received from the University of Bonn’s Institute of Crop Science and Resource Conservation (INRES).

### Illumina sequencing and quality control

TRIzol reagent kit (Catalog # 12183555, Thermofisher) was used to extract total RNA from root tissues of wheat cultivars. The NanoDropTM 1000 spectrophotometer (Thermo Scientific®) was used to determine the quality and amount of RNA. RNA samples were sequenced from commercial company (GenXPRo Frankfurt, Germany). Subsequently, paired end (PE) RNA-Seq libraries were prepared, and RNA sequencing was performed using Illumina NGS HiSeq2000 platform. Number of reads obtained per lane was significantly high, ranging from 10.5 to 13.3 million per sample with average reads per sample was around 12 million. Reads were 100 nt in length. Trimmomatic-0.33 [29] was used with default parameters for trimming. The FastQC quality control tool [30] was used for assessment of quality of reads.

RETRACTED

### Detection of RNA editing site (RES)

All potential RES were calculated with the help of SPRINT (https://sprint.tianlab.cn/, SnP-free RNA editing Identification Toolkit) by using default setting [31]. To support the prediction, we used the SNP calling tool GATK [32] to analyze the mapping BAM files and detect the SNP between RNA sequence and reference genomic DNA (ftp://ftp.ensemblgenomes.org/pub/release-25/plants/fasta/triticum_aestivum/dna/). The overlapped data from both methods were kept for further investigation. The editing sites were then further filtered using the following criteria: (1) editing reads to total mapped reads ratio greater than 50; (2) edited sites with more than five mapped reads. The Ensemble Variant Effect Predictor (VEP) tool (https://asia.ensembl.org/info/docs/tools/vep/index.html) with default parameters was used to annotate the RNA editing site [33].

### Expression analyses of RNA editing gene families

Using transcriptome analysis of RNA-seq data, the levels of gene expression of the *PPR* (*pentatricopeptide repeat*), *OZ1* (*organelle zinc-finger*), and *RIP (RNA editing factor interacting proteins*) gene families in wheat were assessed and compared using NOIseq package. The protein sequences of *Triticum aestivum* PPR, OZ1, and Multiple organellar RNA editing factor (MORF)/ RIP were obtained from the Ensembl database [34]. The procedure reported in our previous work was employed for transcriptome analysis [35]. In details, total RNA from root samples of wheat genotypes was extracted using Gene JET™ Plant RNA Purification Mini Kit (Catalog # K0801). Paired end (PE) sequencing was done with Illumina HiSeq2500 platform. FastQC (http://www.bioinformatics.bbsrc.ac.uk/projects/fastqc/) was used for quality checking and Trimmomatic tool was also used for trimming of reads (quality scores < 20, reads with ambiguous “N” bases more than 10% bases, and reads with less than 15 bases were also trimmed). NOIseq package [36] was used to calculate the FPKM (Fragments per kilobase per million) values. PPR, OZ1, and MORF/RIP proteins expression values were also normalized, and a heatmap was displayed for all genes using the “pheatmap” tool in R [37].

RETRACTED

### Quantitative RT-PCR assay

qRT-PCR tests were used to examine the expression of the *PPR*, *RIP*, and *OZ1* gene families in roots of wheat under the same condition used for RNA-Seq analysis. qRT-PCR studies were done using a Step One Plus Real-Time PCR System (Applied Biosystems, Foster City, CA, USA) using SYBR Premix Ex Taq (Tli RNaseH Plus, Catalog # RR420A) and a Prime Script RT reagent Kit with gDNA Eraser (Takara, Otsu, Japan, Catalog # RR047B). To standardize the expression data, the wheat gene *RLI* (RNase L inhibitor-like protein) was used as an internal control [38]. The 2-ΔΔCt technique was used to assess gene expression [39, 40]. Three biological replicates were used for each gene. Gene-specific primers are enlisted in S1 File.

## Results

### Assessment of RNA-seq data

Total RNA from roots was collected and sequenced using the Illumina HiSeq 2500 platform to gain a better understanding of drought-sensitive and drought-tolerant genotypes. The quality control of raw reads was checked to detect sequencing errors by analyzing sequence quality, GC percentage, the adaptors sequences, and duplicated reads (S2 File). The accuracy of a sequence was assessed using the Phred quality score (Q-score >20). For all genotypes, the value of Q20 was greater than 98%, whereas the value of Q30 was greater than 92%. S2 File shows that the sequencing was done with great precision. All genotypes had average of 48% of GC values. For further downstream analysis, the mean Phred score was within acceptable range. A total of 48.6, 48.5, 48.4, 52.4, 50.4, and 50.6 million clean reads were obtained for Batis, Blue Silver, Chakwal 50, Local White, Syn-22, and UZ-11-CWA-8, respectively. After trimming, an average of 47, 46, 46, 50, 48, and 49 million clean reads were obtained for Batis, Blue Silver, Chakwal 50, Local White, Syn-22, and UZ-11-CWA-8, respectively.

### RNA editing sites prediction in wheat genotypes

The levels of stringency employed to reduce false positives affect the computational detection of RNA editing by RNA seq. This is especially true when using transcriptome data only [41]. Only RNA-seq data can be used to identify RNA-editing sites at the full transcriptome level.

Total identified RESs in Batis were 15032, out of which 3770 were presented on 749 protein coding genes and *TraesCS1D02G346400* has maximum 21 RESs and RNA-editing sites were discovered utilizing the methods mentioned above [42]. There are 44 RESs detected on 9 non protein coding genes (Fig 1). In Blue Silver, total identified RESs were 15183, out of which 3727 were presented on 727 protein coding genes. *TraesCS1A02G353700* and *TraesCS2D02G564600* have maximum 19 RESs. There were 30 RESs detected on 7 non protein coding genes (Fig 1). Chromosome 2B have highest number of edited genes and 6A chromosome have lowest number of edited genes in Batis and Blue Silver. Total identified RESs in Chakwal 50 were 13325, out of which 3658 were presented on 740 protein coding genes and *TraesCS1D02G264200* has maximum 16 RESs. There were 38 RESs detected on 8 non protein coding genes. Chromosome 1B have highest number of edited genes and 7B chromosome have lowest number of edited genes (Fig 1). Total identified RESs in Local White were 17298, out of which 4744 were presented on 950 protein coding genes and *TraesCS4A02G440000* has maximum 19 RESs. There were 9 RESs detected on 2 non protein coding genes. Chromosome 5B have highest number of edited genes and 4B chromosome have lowest number of edited genes (Fig 1). Total identified RESs in Syn-22 were 16680, out of which 4105 were presented on 814 protein coding genes, *TraesCS2B02G225200* and *TraesCS3D02G446700* have maximum 15 RESs. There were 31 RESs detected on 7 non protein coding genes. Chromosomes 2B and 5D have highest number of edited genes and 6A chromosome have lowest number of edited genes (Fig 1). Total identified RESs in UZ-11-CWA-8 were 15596, out of which 3852 were presented on 786 protein coding genes and *TraesCS1A02G188600* has maximum 18 RESs. There are 9 RESs detected on 2 non protein coding genes. Chromosome 2B have highest number of edited genes and 4B chromosome have lowest number of edited genes (Fig 1). The 439, 430, 445, 611, 498, 512 are uniquely identified genes in Batis, Blue Silver, Chakwal 50, Local White, Syn-22, and UZ-11-CWA-8, respectively, in which RESs were predicted. The results indicate that Local White owned the highest unique sites, with the number of 14163, followed by Syn-22, UZ-11-CWA-8, Batis, Blue Silver, and Chakwal 50 with the numbers of 13858, 13385, 12101, 11813, and 10793, respectively (Fig 1). RESs appear on each chromosome, emphasizing the widespread nature of RESs (Fig 2).

RETRACTED

**Fig 1:** Abundance of RNA editing events by Venn diagram analysis among six genotypes of wheat. The genotypes (Blue Silver = light yellow; Syn-22 = light blue; Chakwal 50 = light grey; UZ-11-CWA-8 = light cyan; Local White = light green; and Batis = light orange) were shown with different colors.

**Fig 2:** Genome wide distribution of RESs. Each circle represents the number of all RESs from outside to inside for Batis (G1), Blue Silver (G2), Chakwal 50 (G3), Local White (G4), Syn-22 (G5), and UZ-11-CWA-8 (G6) genotypes.

### Distribution of RNA editing (RE) types

RNA editing is a critical tool for enhancing genetic information and guiding several biological activities after transcription. In this study, Batis was found to have 11 different forms of RNA editing: A-to-G, A-to-C, A-to-T, C-to-A, C-to-G, C-to-T, G-to-A, G-to-C, G-to-T, T-to-A, T-to-C, and T-to-G of which A-to-G and T-to-C editing types were significantly higher than the other types, accounting for up to 27.85% and 26.90%, respectively, of the identified RNA editing sites. Any A-to-C conversion in Batis transcriptome was not detected while percentage of C-to-A, G-to-C, T-to-A, G-to-T, C-to-G, and T-to-G substitution was less than 1 (Fig 3). In Blue Silver genotype, 10 types of RNA editing were noticed: A-to-G, A-to-T, C-to-G, C-to-T, G-to-A, G-to-C, G-to-T, T-to-A, T-to-C, and T-to-G of which A-to-G and T-to-C editing types were significantly higher than the other types, accounting for up to 24% and 25.49%, respectively, of the identified RNA editing sites. Any A-to-C, C-to-A conversion in Blue Silver transcriptome was not detected while percentage of C-to-G, G-to-C, G-to-T, and T-to-G substitution was less than 1 (Fig 3).

**Fig 3:** The frequency of different types of nucleotides editing events in whole transcriptome of six genotypes of wheat.

In Chakwal 50, 11 types of RNA editing were detected, including possible base substitutions as follows: A-to-G, A-to-T, C-to-A, C-to-G, C-to-T, G-to-A, G-to-C, G-to-T, T-to-A, T-to-C, and T-to-G of which A-to-G and T-to-C editing types were significantly higher than the other types, accounting for up to 25% and 25.41%, respectively. Any A-to-C conversion in Chakwal 50 transcriptome was not detected, while percentage of C-to-A, C-to-G, G-to-C, G-to-T and T-to-G substitution was less than 1 (Fig 3). Similarly in Local White, 12 types of RNA editing were noticed: A-to-C, A-to-G, A-to-T, C-to-A, C-to-G, C-to-T, G-to-A, G-to-C, G-to-T, T-to-A, T-to-C, and T-to-G of which A-to-G, T-to-C and C-to-T editing types were significantly higher than the other types, accounting for up to 25.28%, 24.35% and 24.69%, respectively, while percentage of A-to-C, A-to-T, C-to-A, C-to-G, G-to-C, G-to-T, T-to-A and T-to-G substitution was less than 1 (Fig 3). Syn-22 also have 12 types of RNA editing: A-to-C, A-to-G, A-to-T, C-to-A, C-to-G, C-to-T, G-to-A, G-to-C, G-to-T, T-to-A, T-to-C, and T-to-G of which A-to-G, G-to-A, T-to-C and C-to-T editing types were significantly higher than the other types, accounting for up to 29.92%, 20.24%, 29.09, and 18.36%, respectively, of the identified RNA editing sites, while percentage of A-to-C, A-to-T, C-to-A, C-to-G, G-to-C, G-to-T, T-to-A and T-to-G substitution was less than 1 (Fig 3). In UZ-11-CWA-8, 10 types of RNA editing were noticed: A-to-G, A-to-T, C-to-A, C-to-G, C-to-T, G-to-A, G-to-C, G-to-T, T-to-A, and T-to-C of which A-to-G and T-to-C editing types were significantly higher than the other types, accounting for up to 26.56% and 28.03%, respectively; of the identified RNA editing sites. Any A-to-C, T-to-G conversion in UZ-11-CWA-8 transcriptome was not detected while percentage of A-to-T, C-to-A, C-to-G, G-to-C, T-to-A, and G-to-T substitution was less than 1 (Fig 3).

RETRACTED

The results indicates Syn-22 have the highest transition rate with number of (A/G = 4991, T/C = 4853) and lowest transversion rate with number of (A/C = 5, A/T = 117, C/G = 72, T/G = 5) followed by Local White with the number of transition (A/G = 4374, T/C = 4213) and transversion (A/C = 5, A/T = 123, C/G = 66, T/G = 5), UZ-11-CWA-8 with the number of transition (A/G = 4143, T/C = 4373) and transversion (A/C = 0, A/T = 124, C/G = 94, T/G = 0), Batis with the number of transition (A/G = 4187, T/C = 4044) and transversion (A/C = 0, A/T = 166, C/G = 86, T/G = 5), Blue Silver with the number of transition (A/G = 3723, T/C = 3871) and transversion (A/C = 0, A/T = 182, C/G = 47, T/G = 5) and Chakwal 50 with the number of transition (A/G = 3339, T/C = 3387) and transversion (A/C = 0, A/T = 139, C/G = 90, T/G = 5), these results are consistent with the previous studies [43, 44].

### Expression analysis of *PPR*, *MORF*/*RIP*, and *OZ1* genes

To figure out why six wheat genotypes had varying numbers of RNA editing? We looked at the expression of three gene (*PPR*, *MORF/RIP*, and *OZ1****)*** families which might be involved in RNA editing process. In wheat, a total of 24, 29, and 278 proteins were identified as OZ1, MORF/RIP and PPR, respectively, by using key words in wheat Ensembl Plants database (https://plants.ensembl.org/Triticum_aestivum/Info/Index). The expression level of these gene families in different type of wheat genotypes were measured by RNA seq. The expression level of most of *OZ1* gene family is higher in Local White, Chakwal 50, UZ-11-CWA-8, and Syn-22 in which higher number of RESs were identified, implying that normal growth conditions for different genotypes might modify RNA editing events and have an impact on gene expression levels in these drought-tolerant genotypes. Expression levels of this gene family by RNA seq in different genotypes of wheat also shown in Fig 4 and expression values in FPKM are listed in S3 File. The expression level of four genes of *OZ1* gene family also determined by qRT-PCR. The expression level of these genes *TraesCS3A02G396300* (*OZ1*), *TraesCS2A02G226400* (*OZ2*), *TraesCS3B02G225200* (*OZ3*), and *TraesCS3B02G370800* (*OZ4*) by qRT-PCR is shown in Fig 5A–5D, and these results are consistent with expression level calculated by RNA seq.

RETRACTED

**Fig 4:** Visualization of differentially expressed genes of *OZ1* (rows) by RNA seq in six genotypes of wheat. Blue indicates low, Brown indicates medium red indicates high expression in heatmap.

**Fig 5:** Measurements of gene expression of *OZ1* by qRT-PCR. The relative gene expression of DEGs by qRT-PCR is represent by bars with standard errors in three independent experiments. Least Significant Difference (LSD) test was used. Different lowercase letters indicate significantly differences at *P* ≤ 0.05.

We also looked at the expression of *MORF*/*RIP* to see why six wheat genotypes had varying numbers of RNA editing? More genes of this family were upregulated in drought-tolerant genotypes identified by RNA-seq data as shown in Fig 6 and their values in FPKM are listed in S4 File. Only one gene *TraesCS5B02G290000* not expressed in any genotype of wheat. The expression level of 4 genes *TraesCS6D02G007100* (*RIP1*), *TraesCS4D02G104800* (*RIP2*), *TraesCS7A02G050200* (*RIP3*), and *TraesCS5B02G289900* (*RIP4*) of this family also noticed by qRT-PCR as shown in Fig 7A–7D.

**Fig 6:** Visualization of differentially expressed genes of *MORF/RIP* (rows) by RNA seq in six genotypes of wheat. Blue indicates low, Brown indicates medium red indicates high expression in heatmap.

**Fig 7:** Measurements of gene expression of *MORF/RIP* by qRT-PCR. The relative gene expression of DEGs by qRT-PCR is represent by bars with standard errors in three independent experiments. Least Significant Difference (LSD) test was used. Different lowercase letters indicate significantly differences at *P* ≤ 0.05.

The levels of gene expression of *PPR* genes in six wheat genotypes were measured and compared using transcriptome analysis of RNA-seq data. However, no significant differences in expression were found for *PPR* genes under normal growth conditions, implying that normal growth conditions solely affect RNA editing events and had no effect on expression levels for this gene family as compared to *OZ1* and *RIP* gene families. Surprisingly, only six *PPR* genes showed a high level of expression across all genotypes, as shown in Fig 8 and S5 File showing the expression values in FPKM. To verify the reliability of RNA-seq, the expression level of four genes *TraesCS6B02G249200 (PPR1)*, *TraesCS6D02G202700 (PPR2)*, *TraesCS5B02G038400 (PPR3)*, and *TraesCS5A02G037400 (PPR4)* from this gene family were determined by qRT-PCR (Fig 9A–9D). The qRT-PCR showed that the expression pattern of these four DEGs was like those found by RNA-seq, confirming the reliability of the sequencing data.

RETRACTED

**Fig 8:** Visualization of differentially expressed genes of *PPR* (rows) by RNA seq in six genotypes of wheat. Blue indicates low, Brown indicates medium red indicates high expression in heatmap.

**Fig 9:** Measurements of gene expression of *PPR* by qRT-PCR. The relative gene expression of DEGs by qRT-PCR is represent by bars with standard errors in three independent experiments. Least Significant Difference (LSD) test was used. Different lowercase letters indicate significantly differences at *P* ≤ 0.05.

### Annotation of RNA editing sites

We used the VEP to annotate the RNA editing sites. Based on genetic characteristics, we classified the RESs into eight groups: All genotypes listed in S6–S11 Files, had intron variants, upstream gene variants, intergenic variants, downstream gene variants, missense variants, 5′-UTR variants, 3′-UTR variants, synonymous variants, stop gained, and others. Results showed that Local White owned the highest (5723) RESs in CDS region of protein coding genes, followed by Chakwal 50 (4528), Batis (4505), Blue Silver (4356), Syn-22 (4031), and UZ-11-CWA-8 (3758). As indicated in S12 File, Blue Silver and Local White have the most RESs in 3´-UTR, while Batis and Syn-22 have the most RESs in 5´-UTR, implying that most RESs may cause changes in protein sequence.

In total, 2466 editing sites in 661 genes were found to result in an amino acid change, with 1 editing event converting a hydrophilic amino acid to a hydrophobic amino acid, 164 converting a hydrophilic amino acid to a neutral amino acid, 291 converting a hydrophobic amino acid to a hydrophilic amino acid, 373 converting a hydrophobic amino acid to a neutral amino acid, and 730 converting a neutral amino acid to a hydrophilic in Batis genotype. Similarly, 2279 editing sites in 624 genes were found to result in an amino acid change, with 86 editing events converting hydrophilic amino acids to hydrophobic amino acids, 157 editing events converting hydrophilic amino acids to neutral amino acids, 17 editing events converting hydrophobic amino acids to hydrophilic amino acids, 285 editing events converting hydrophobic amino acids to hydrophilic amino acids, and 285 editing events converting hydrophobic amino acids to hydrophilic amino acids in Blue Silver. In Chakwal 50, there were 2413 editing sites in 662 genes that resulted in amino acid change, with 135 editing events converting hydrophilic amino acids to hydrophobic amino acids, 124 editing events converting hydrophilic amino acids to neutral amino acids, 52 editing events converting hydrophobic amino acids to hydrophilic amino acids, and 327 editing events converting hydrophobic amino acids to neutral amino acids. Totally, 3129 editing sites in 846 genes were observed to result in the amino acid change, of which 154 editing events led to a conversion from hydrophilic amino acid to hydrophobic amino acid, 180 changing from hydrophilic amino acid to neutral amino acid, 14 changing from hydrophobic amino acid to hydrophilic amino acid, 394 changing from hydrophobic amino acid to neutral amino acid, 359 changing from neutral amino acid to hydrophilic amino acid and 398 changing from neutral amino acid to hydrophobic amino acid in Local White. Totally, 2124 editing sites in 547 genes were observed to result in the amino acid change, of which 103 editing events led to a conversion from hydrophilic amino acid to hydrophobic amino acid, 131 changing from hydrophilic amino acid to neutral amino acid, 11 changing from hydrophobic amino acid to hydrophilic amino acid, 286 changing from hydrophobic amino acid to neutral amino acid, 401 changing from neutral amino acid to hydrophilic amino acid and 398 changing from neutral amino acid to hydrophobic amino acid in Syn-22. Totally, 1902 editing sites in 530 genes were observed to result in the amino acid change, of which 96 editing events led to a conversion from hydrophilic amino acid to hydrophobic amino acid, 83 changing from hydrophilic amino acid to neutral amino acid, 18 changing from hydrophobic amino acid to hydrophilic amino acid, 293 changing from hydrophobic amino acid to neutral amino acid, 232 changing from neutral amino acid to hydrophilic amino acid and 333 changing from neutral amino acid to hydrophobic amino acid in UZ-11-CWA-8 as shown in S13 File. Green, blue, and red colors are used to show the hydrophilic, hydrophobic, and neutral amino acids, respectively. The above results were in good agreement with previous studies [45, 46], which demonstrated that the RNA editing caused an overall increase in hydrophobicity of the resulting proteins.

RETRACTED

### Identification of A-to-I RNA editing

In Batis genotype, total of the 2952 A-to-I RESs were identified in which 1462 A-to-G RESs and 1490 T-to-C RESs. In A-to-I RESs, 2775 hyper-RES were identified that was higher than 182 regular-RES. 437 A-to-I editing types were associated with 74 protein encoding genes. In Blue Silver, total identified A-to-I RESs were 2977, out of which 1446 are A-to-G and 1531 are T-to-C. 270 A-to-I editing type were associated with 52 protein encoding genes. In Chakwal 50, total identified A-to-I RESs were 1916, out of which 884 were A-to-G and 1032 were T-to-C. 259 A-to-I editing types were associated with 52 protein encoding genes. In Local White, total identified A-to-I RESs were 2576, out of which 1305 were A-to-G and 1271 were T-to-C. 244 A-to-I editing type were associated with 50 protein encoding genes. In Syn-22, total identified A-to-I RESs were 3422, out of which 1750 were A-to-G and 1672 were T-to-C. 244 A-to-I editing type were associated with 49 protein encoding genes. In UZ-11-CWA-8, total identified A-to-I RESs were 3459, out of which 1641were A-to-G and 1818 were T-to-C. 375 A-to-I editing type were associated with 64 protein encoding genes. Gene Ontology (GO) term also find and mostly genes involved in nitrogen compound metabolic process as shown in S14 File.

### GO analysis of protein coding genes associated with RESs

To determine the functions of the genes in which RNA editing site was detected in this study, all REGs in each genotype were annotated to the terms in the GO database. Results showed that 26, 23, 21, 18, 26, and 20 significantly enriched molecular functions identified in Batis, Blue Silver, Chakwal 50, Local White, Syn-22, and UZ-11-CWA-8, respectively. The most enriched terms identified in each genotype are as energy derivation by oxidation of organic compounds, nucleosome organization, chromatin assembly, DNA packaging, aerobic electron transport chain, DNA conformation change, protein-DNA complex subunit organization, ATP synthesis coupled electron transport, oxidative phosphorylation, electron transport chain, ATP metabolic process, amide biosynthetic process, response to water deprivation, protein-DNA complex assembly, respiratory electron transport chain, cellular amide metabolic process, heat shock protein binding, response to water, peptide metabolic process, response to inorganic substance and peptide biosynthetic process and proline dehydrogenase activity as shown in S15 File.

## Discussion

RNA editing is the epigenetic machinery that causes deletions, insertions, and substitutions in transcripts, as well as the increase of the transcriptome’s complexity through the diversification of genomically encoded information. It was reported in Kinetoplastid protozoa and many species [47]. RNA editing process is engaged in a variety of biological processes; for example, disrupting intron structures can increase RNA splicing [48, 49]. It also affects the functions of microRNA (miRNA) and RNA degradation. Plant development and evolutionary adaption are both aided by RNA editing of gene transcripts. Variation in RESs at a specific position in mitochondrial genes can have a deleterious impact on plant growth, fertility, development, and seed development [12, 50–52]. Some studies also suggests that RNA editing involved in plant adaptation to environmental stress conditions (e.g., UV, severe temperatures, and oxidative stress) and has consequences during evolution [53, 54]. In addition, some data suggests that environmental conditions, such as cold stress in rice and heat stress in maize influence RNA editing [55, 56]. Before the next generation sequencing, the RESs was identified by comparing RT-PCR results to the genomic DNA sequence this method is sluggish and prone to overestimate editing level.

RETRACTED

RNA-seq is a powerful technique for identifying all possible RNA editing sites and quantifying their editing extent, particularly for sites with low editing extent. As a result, with the introduction of sequencing technology, RNA sequencing is now utilized to find RESs in numerous organisms [57–59]. The 12 different types of RESs found in non-coding regions including the 3′-UTR and 5′-UTR, rRNA, Upstream and downstream of genes, tRNAs, and translated regions (S12 File). RNA editing sites are widely found in protein-coding regions, causing alterations in protein structure and function [9, 20, 60]. We found hundreds of RNA editing sites across all genotypes and provide a useful data set for future researchers. These RESs not been reported previously. In certain circumstances, RNA editing responsible for amino acid changes is required for functional protein production, but there are a few exceptions: plants still demonstrate site editing even if the encoded protein’s function is not required. RNA editing can occur at the first, second, or third codon positions in protein-coding regions, resulting in changes in physicochemical properties of amino acid [2]. We also discovered that the modifications in amino acids tend to be hydrophobic, hydrophilic, and neutral, which is consistent with earlier research (S13 File). In plants, RNA editing serves as an extra proofreading mechanism for correcting DNA mutations at the RNA level in order to achieve protein functionalities [9, 45, 61]. RNA editing has been involved in architectural growth, regulating organ formation, and development in various studies [7, 62–64]. RESs in intronic and UTRs regions of genes may affect mRNA stability and splicing [49, 65–67], we also detect the RESs in intronic and UTRs regions of genes. Our results showed that the transition rate is higher than transversion. In animals, the transition rate is also higher as compared to transversion. Transversion is a complicated process and might have negative effects [68]. Our results showed higher number of RESs in drought-tolerant genotypes in comparison to drought-sensitive genotypes. This makes drought-tolerant genotypes more adaptive to environmental stress.

RETRACTED

This conclusion is in line with previous research that demonstrated RESs controls plant development, organ formation, growth in the stress condition [69, 70]. In Local White, Syn-22, and UZ-11-CWA-8 genotypes, more RESs has predicted followed by Batis, Blue Silver, and Chakwal 50. Furthermore, we determined the higher number of RESs in the drought-tolerant genotypes altered the expression of numerus genes involved in the deeper root system and metabolism of many organic macromolecules. The editing resulted in a stop coding or amino acid alteration, which is consistent with empirical facts indicating RNA processing occur and implying that RNA editing could be a key regulator in the activation of drought tolerance systems and pathways. The environmental stress such as temperature, soil nutrients, soil texture, and metal ion concentration have the direct effect on RNA in cells and act as a sensor [71]. The results showed that the thermo-sensitive secondary and tertiary structures of RNA cause higher rate of transition and RESs in drought-tolerant genotypes. *PPR* gene family has been identified in many plant species such as *Arabidopsis thaliana* and *Oryza sativa*, and involved in RNA processing [54, 72]. According to our finding, the expression of most PPR proteins was dramatically higher in drought-tolerant genotypes. Previously also reported that *OZ1* binds to *RIP* protein and interact with *PPR* [73]. Our results also explained that the expression of *OZ1* and *RIP* is also higher in drought-tolerant genotypes. This makes them more adaptive to environmental stress. Despite this, one *PPR* member in any genotypes of wheat was not expressed, this gene may have specific role in drought-tolerant genotypes. Further effort needs to be put into clarify their involvement (or not) in RNA editing.

## Conclusion

In this study, we systematically identified the RNA editing sites (RESs) in roots tissue of wheat and checked the gene expression analysis of *OZ1*, *PPR1*, and *RIP* gene families in drought-tolerant and susceptible genotypes. More RESs were detected in drought-tolerant as compare to drought-susceptible genotypes. RNA editing not only controls plant organ formation and development but also plays an indispensable role in response to diverse environment conditions and suggesting that RNA editing might act as a “regulator” to control the root architecture development. Furthermore, the regulatory network of the essential genes in which RESs were detected were investigated. Nitrogen compound metabolic process and phytohormone signal transduction might play important role in roots development which helps wheat plant adaptation to harsh climatic conditions. These findings will contribute to improve understanding the molecular mechanism of dynamics of gene regulation in root architecture development in wheat at posttranscriptional level.

RETRACTED

## Supporting information

S1 File List of primers sequences used for qRT-PCR analysis. (XLSX)

S2 File Basic statistics of total raw and clean reads of six genotypes. (XLSX)

S3 File Expression level of *OZ1* gene family in six types of wheat genotype. (XLSX)

S4 File Expression level of *MORF/RIP* gene family in six types of wheat genotype. (XLSX)

S5 File Expression level of *PPR* gene family in six types of wheat genotype. (XLSX)

S6 File Characterization of RESs in Batis. (XLSX)

S7 File Characterization of RESs in Blue Silver. (XLSX)

S8 File Characterization of RESs in Chakwal 50. (XLSX)

S9 File Characterization of RESs in Local White. (XLSX)

S10 File Characterization of RESs in Syn-22. (XLSX)

S11 File Characterization of RESs in UZ-11-CWA-8. (XLSX)

S12 File Basic annotation of editing sites in six genotypes of wheat. (XLSX)

S13 File The change type among hydrophilic amino acid, hydrophobic amino acid, and terminator due to RNA editing. (XLSX)

S14 File Function annotation of genes in which A-to-I RESs predicted. (XLSX)

S15 File Gene ontology of genes in six wheat genotypes. (XLSX)
